RETRACTED

# Application Value of NT-proBNP Combined with NLR in Evaluation of Major Adverse Cardiac Events in Elderly Patients with Chronic Heart Failure

**DOI:** 10.1155/2022/3689445

**Published:** 2022-10-14

**Authors:** Zhiyong Li, Hui Rong, Wenxun Wu, Ting Huang, Jun Xu

**Affiliations:** ^1^Department of Geriatrics, General Hospital of Pingxiang Mining Group Company with Limited Liability, Pingxiang 337035, Jiangxi, China; ^2^Department of Internal Medicine-Cardiovascular, General Hospital of Pingxiang Mining Group Company with Limited Liability, Pingxiang 337035, Jiangxi, China; ^3^Clinical Laboratory, General Hospital of Pingxiang Mining Group Company with Limited Liability, Pingxiang 337035, Jiangxi, China; ^4^Department of Hematology, General Hospital of Pingxiang Mining Group Company with Limited Liability, Pingxiang 337035, Jiangxi, China

## Abstract

**Objective:**

To explore the application value of N-terminal pro-B type natriuretic peptide (NT-proBNP) combined with neutrophil-to-lymphocyte ratio (NLR) in evaluation of major adverse cardiac events (MACEs) in elderly patients with chronic heart failure (CHF).

**Methods:**

50 CHF patients admitted to the Department of Cardiovascular Medicine of our hospital from January 2021 to December 2021 were selected as the observation group. Another 50 non-CHF patients of our hospital were selected as the control group. Clinical data were collected from subjects who met the inclusion criteria, including general information, personal disease history, and laboratory test indicators. Patients with CHF were followed up for 6 months. Patients with CHF were divided into two groups, MACE group and non-MACE group.

**Results:**

The levels of WBC, NEU, NLR, and NT-proBNP in observation group were higher than those in control group, but the level of LYM was the opposite (*P* < 0.05). The age, WBC, NEU, LYM, PLT, blood glucose, NLR, and NT-proBNP of MACE group and non-MACE group were significantly different (*P* < 0.05). The increased levels of NEU, NLR, NT-proBNP and the decreased levels of LYM and PLT are all independent risk factors for MACE in elderly patients with CHF (*P* < 0.05). The AUC of NLR in evaluating the occurrence of MACE in elderly CHF patients was 0.841. When the Youden index was 0.7692, the sensitivity was 76.92% and the specificity was 100.00%. The AUC of NT-proBNP in evaluating the occurrence of MACE in elderly CHF patients was 0.705. When the Youden index was 0.5260, the sensitivity was 76.92% and the specificity was 75.68%. The AUC of NT-proBNP combined with NLR in evaluating the occurrence of MACE in elderly CHF patients was 0.954. When the Youden index was 0.8420, the sensitivity was 92.31% and the specificity was 91.89%.

RETRACTED

**Conclusion:**

NT-proBNP combined with NLR has high value in the evaluation of MACE in elderly CHF patients and can be used as an auxiliary predictive index in clinic.

## 1. Introduction

Chronic heart failure (CHF) is a serious stage of many cardiovascular diseases, mainly caused by hypertension, coronary heart disease, myocardial ischemia, stress response, cardiac insufficiency, and other inducements [1]. The pathogenesis of CHF is complex, and the common clinical symptoms are dyspnea, limited exercise tolerance, chest tightness, shortness of breath, lower limb edema, and fatigue [2]. Studies have shown that the onset of CHF is mainly in the elderly, and the elderly patients with CHF are usually older than 70 years [3]. For the elderly, this population is often accompanied by a variety of diseases, so the clinical symptoms and signs of CHF patients are atypical, and it is difficult to get effective treatment in time, thus increasing the mortality of patients [4]. CHF can damage patients' health status and bring heavy medical and health care burden to patients and their families. At present, the global aging trend is getting worse, and CHF has gradually become one of the public health problems that threaten people's lives and health [5]. The prognosis of elderly patients with CHF is mainly related to long-term progressive underlying diseases, myocardial injury, heredity, environment, and other factors. Among them, the most common poor prognosis for patients with CHF is the main adverse cardiac event (MACE), which is the main cause of disability and death in patients with CHF and seriously reduces the quality of life of their patients [6, 7]. Therefore, it is necessary to predict the sensitive indicators of MACE in elderly CHF patients clinically, which is especially important to improve people's prognosis.

N-terminal pro-B type natriuretic peptide (NT-proBNP) is an inactive N-terminal fragment of probrain natriuretic peptide (BNP) hormone after splitting, which has the characteristics of longer half-life and more stability [8]. As a natural hormone synthesized by cardiac myocytes, NT-proBNP has attracted increasing attention in evaluating the severity and prognosis of CHF [9]. In addition, inflammatory factors are also involved in the pathogenesis, disease progression, and prognosis of CHF in a variety of ways. CHF patients are often accompanied by abnormal release of proinflammatory factors and aggravation of systemic inflammatory response [10]. Neutrophil-to-lymphocyte ratio (NLR), as a common inflammatory marker, can indicate the ratio of neutrophil (NEU) to lymphocyte (LYM), which has become a research hotspot of cardiologists [11].

RETRACTED

At present, there are few reports about the evaluation value of NT-proBNP combined with NLR in elderly CHF patients with MACE. We will analyze this content in order to improve the prognosis of patients.

## 2. Data and Methods

### 2.1. General Information

50 CHF patients admitted to the Department of Cardiovascular Medicine of our hospital from January 2021 to December 2021 were selected as the observation group. Inclusion criteria are as follows: the age ranged from 65-82 years, with an average age of (74.16 ± 2.94) years; all patients met the 2016 ESC Guidelines for the diagnosis and treatment of acute and chronic heart failure [12]; NYHA is classified as II-IV; and all patients were treated according to the 2016 ESC Guidelines. Exclusion criteria are as follows: accompanied by chronic obstructive pulmonary disease, pulmonary interstitial fibrosis, primary pulmonary hypertension, nonthrombotic disease, chronic kidney disease, liver cirrhosis, venous insufficiency, acute myocardial infarction, severe arrhythmia, malignant tumor, blood system disease, infections, and other diseases that affect white blood cell counts; patients with missing case data; and patients who died due to non-MACE factors during the follow-up period. Another 50 non-CHF patients of our hospital were selected as the control group.

### 2.2. Research Methods

Clinical data were collected from subjects who met the inclusion criteria, including general information (age and sex), personal disease history (coronary heart disease, diabetes, and hypertension), and laboratory examination indicators (white blood cell (WBC), NEU, LYM, platelet count (PLT), blood glucose, NLR, and NT-proBNP).

Patients with CHF were followed up for 6 months, and the follow-up mode was outpatient follow-up or telephone. The end point of follow-up was MACE or death. MACE includes cardiac death, nonfatal myocardial infarction, and hospitalization for recurrent heart failure. Patients with CHF were divided into MACE group and non-MACE group according to the occurrence of MACE.

### 2.3. Statistical Methods

SPSS 22.0 software was used for processing, and the measurement data were expressed as mean ± standard deviation ($\bar{x}$ ± *s*), and *t*-test was used for comparison. The data are expressed as %, and the comparison was made by *χ*^2^ test. Logistic regression was used to analyze the influencing factors of MACE. ROC was used to analyze the evaluation value of different indexes on the occurrence of MACE. *P* < 0.05 was statistically significant.

## 3. Results

### 3.1. Comparison of Clinical Data between Observation Group and Control Group

The levels of WBC, NEU, NLR, and NT-proBNP in the observation group were higher than those in the control group, but the level of LYM was the opposite (*P* < 0.05) (see Table 1).

RETRACTED

### 3.2. Comparison of Clinical Data between MACE Group and Non-MACE Group

There were 13 CHF patients with MACE in the observation group. The age, WBC, NEU, LYM, PLT, blood glucose, NLR, and NT-proBNP of the MACE group and non-MACE group were significantly different (*P* < 0.05) (see Table 2).

### 3.3. Multivariate Analysis of MACE in Elderly CHF Patients

Age, white blood cells, NEU, LYM, platelets, blood sugar, NLR, and NT-proBNP were assigned according to the average of all CHF patients. See Table 3 for the assignment. The increased levels of NEU, NLR, and NT-proBNP and the decreased levels of LYM and PLT are all independent risk factors for MACE in elderly patients with CHF (*P* < 0.05) (see Table 4).

### 3.4. ROC of MACE in Elderly CHF Patients was Assessed by Different Indicators

The AUC of NLR in evaluating the occurrence of MACE in elderly CHF patients was 0.841. When the Youden index was 0.7692, the sensitivity was 76.92% and the specificity was 100.00%. The AUC of NT-proBNP in evaluating the occurrence of MACE in elderly CHF patients was 0.705. When the Youden index was 0.5260, the sensitivity was 76.92% and the specificity was 75.68% (see Table 5 and Figure 1).

### 3.5. NT-proBNP Combined with NLR to Evaluate ROC Curve of MACE in Elderly CHF Patients

The AUC of NT-proBNP combined with NLR in evaluating the occurrence of MACE in elderly CHF patients was 0.954. When the Youden index was 0.8420, the sensitivity was 92.31% and the specificity was 91.89% (see Figure 2).

## 4. Discussion

In recent years, good clinical progress has been made in the diagnosis and treatment of CHF. However, due to various factors, the prognosis of CHF patients has not been comprehensively improved, and the risk of MACE after the patient is discharged from hospital is still high [13]. Especially in the elderly patients with CHF, due to the gradual failure of the organs of the elderly, the systolic and diastolic function of the heart is obviously decreased, which leads to the higher incidence of MACE in elderly CHF patients after discharge than in young patients, and higher incidence of disability and death after MACE [14, 15]. Therefore, it is very important to use effective indicators to evaluate the prognosis of elderly CHF patients.

As a metabolite of BNP, NT-proBNP has a relatively stable activity in normal people [16]. Patients with CHF often have ventricular remodeling and cardiac insufficiency after onset, which leads to the increase of atrial pressure, stimulates the release of BNP from the myocardium of atrial wall, and makes BNP rapidly synthesized and released into the blood, which leads to the increase of NT-proBNP level in patients [17]. Schmitt's team found that NT-proBNP can replace the clinical results of heart failure trials and provide higher predictive value for cardiac insufficiency [18]. NEU is one of the most abundant leukocyte types and is involved in active nonspecific inflammation. In the process of inflammation, abnormally high activation of NEU leads to the release of multiple proinflammatory factors and proteolytic enzymes, which amplify the inflammatory response and destroy the cardiomyocytes, causing direct damage to the heart function [19, 20]. LYM is related to physiological stress and plays an important role in inflammation. In CHF patients, the decrease of LYM proliferation and differentiation, inhibition of neurohumoral priming, and LYM apoptosis lead to the decrease of LYM level in patients [21, 22]. NLR, as a compound inflammatory marker of NEU and LYM, can reflect the evaluation characteristics of NEU and LYM at the same time, reflect the sympathetic nerve excitation, and better reflect the systemic inflammatory state, which is of great significance for the evaluation of the condition and prognosis of patients with CHF [23]. Durmus's team studied 56 HF patients and found that compared with non-HF patients, the NLR level of HF patients was improved, and NLR could be used to predict the mortality of HF patients [24]. In this study, compared with the non-CHF population, the levels of NLR and NT-proBNP in elderly CHF patients are higher; compared with the non-MACE group, the levels of NLR and NT-proBNP in the MACE group were higher. In addition, multivariate analysis showed that the increase in level of NLR and NT-proBNP were independent risk factors of MACE in elderly CHF patients. It is suggested that the levels of NLR and NT-proBNP may reflect the prognosis of CHF patients.

RETRACTED

ROC analysis in this study further showed that the AUC of NLR and NT-proBNP in evaluating MACE in elderly CHF patients was 0.841 and 0.705, respectively. The results indicate that NLR and NT-proBNP have certain value in predicting MACE in elderly CHF patients. The detection of NLR has the advantages of simple operation, easy access, low cost, saving detection time, etc., and the variability in the detection process is small [25]. The advantages of NT-proBNP detection are lower detection cost and better prediction effect [26]. However, only using NLR or NT-proBNP to predict the incidence of MACE in elderly patients with CHF is vulnerable to factors such as age, infection, and renal function, and single-index detection still has certain limitations. Therefore, using the combination of the two as an evaluation index for predicting the occurrence of MACE can significantly improve the limitation of single-index detection. We found that the AUC of NT-proBNP combined with NLR in evaluating MACE in elderly CHF patients was higher than that of single index. It shows that the combination of the two has higher value in the prognosis evaluation of elderly CHF patients and can be used as an auxiliary predictive index in clinic.

## 5. Conclusion

To sum up, NT-proBNP combined with NLR has high value in the evaluation of MACE in elderly CHF patients and can be used as an auxiliary predictive index in clinic. This study only selected elderly patients with CHF, and it was a single-center and small-sample study. We need to further improve the research scheme in the future.

## Figures and Tables

**Figure 1:** ROC of MACE in elderly CHF patients was assessed by different indicators (the closer the curve is to the upper left corner of the picture, the higher the prediction value will be. If the curve is lower than the reference line area, it means that the indicator has no prediction significance).

**Figure 2:** ROC curve of NT-proBNP combined with NLR in evaluating MACE in elderly CHF patients.

**Table 1:** Comparison of clinical data between observation group and control group (*n*, $\bar{x}$ ± *s*, %).

Item	Control group (*n* = 50)	Observation group (*n* = 50)	*χ* ^2^/*t* value	*P*-Value
Age (years)	73.54 ± 2.92	74.16 ± 2.94	1.058	0.293
Male	27 (54.00%)	30 (60.00%)	0.367	0.545
History of coronary heart disease	24 (48.00%)	28 (56.00%)	0.641	0.423
History of diabetes	12 (24.00%)	15 (30.00%)	0.457	0.499
History of hypertension	29 (58.00%)	31 (62.00%)	0.167	0.683
WBC (×10^9^/L)	5.77 ± 1.16	6.38 ± 1.34	2.433	0.017
NEU (×10^9^/L)	3.41 ± 0.93	4.88 ± 1.20	6.846	<0.001
LYM (×10^9^/L)	1.95 ± 0.41	1.49 ± 0.28	6.551	<0.001
PLT (×10^9^/L)	202.64 ± 42.72	187.97 ± 39.08	1.791	0.076
Blood glucose (mmol/L)	5.75 ± 1.23	6.20 ± 1.44	1.680	0.096
NLR	1.72 ± 0.16	3.50 ± 1.78	7.043	<0.001
NT-proBNP (pg/ml)	267.34 ± 37.61	3748.11 ± 413.52	59.275	<0.001

**Table 2:** Comparison of clinical data between the MACE group and non-MACE group (*n*, $\bar{x}$ ± *s*, %).

Item	Non-MACE group (*n* = 37)	MACE group (*n* = 13)	*χ* ^2^/*t* value	*P-*Value
Age (years)	73.59 ± 2.51	75.77 ± 3.54	2.412	0.020
Male	22 (59.46%)	8 (61.54%)	0.017	0.895
History of coronary heart disease	21 (56.76%)	7 (53.85%)	0.033	0.856
History of diabetes	11 (29.73%)	4 (30.77%)	0.005	0.944
History of hypertension	22 (59.46%)	9 (69.23%)	0.390	0.532
WBC (×10^9^/L)	6.12 ± 1.13	7.11 ± 1.66	2.393	0.021
NEU (×10^9^/L)	4.65 ± 1.02	5.55 ± 1.48	2.422	0.019
LYM (×10^9^/L)	1.61 ± 0.21	1.16 ± 0.19	6.802	<0.001
PLT (×10^9^/L)	180.51 ± 33.03	209.23 ± 47.98	2.386	0.021
Blood glucose (mmol/L)	5.92 ± 1.22	6.99 ± 1.78	2.402	0.020
NLR	2.93 ± 0.64	5.12 ± 2.81	4.497	<0.001
NT-proBNP (pg/ml)	3669.08 ± 349.48	3973.06 ± 507.73	2.386	0.021

RETRACTED

**Table 3:** Multifactor assignment.

Item	Coefficient of regression
Age	“<74.16” = “0”; ≥74.14” = “1”
WBC	“<6.38” = “0”; “≥6.38” = “1”
NEU	“<4.88” = “0”; “≥4.88” = “1”
LYM	“≥1.49” = “0”; “<1.49” = “1”
PLT	“≥187.97” = “0”; “<187.97” = “1”
Blood glucose	“<6.20” = “0”; “≥6.20” = “1”
NLR	“<3.50” = “0”; “≥3.50” = “1”
NT-proBNP	“<3748.11” = “0”; “≥3748.11” = “1”

**Table 4:** Multivariate analysis of MACE in elderly CHF patients.

Item	Coefficient of regression	Standard error	Wald value	*P*-Value	OR value	95%CI
Age	0.199	0.150	1.760	0.073	1.220	0.909-1.637
WBC	0.315	0.245	1.653	0.074	1.370	0.847-2.214
NEU	0.406	0.204	3.961	0.041	1.501	1.006-2.238
LYM	0.457	0.186	6.036	0.035	1.579	1.096-2.274
PLT	0.280	0.133	4.432	0.037	1.323	1.019-1.717
Blood glucose	0.332	0.218	2.319	0.059	1.394	0.909-2.136
NLR	0.489	0.164	8.890	0.019	1.631	1.182-2.248
NT-proBNP	0.295	0.101	8.531	0.020	1.343	1.102-1.637

**Table 5:** ROC of MACE in elderly CHF patients was assessed by different indicators.

Item	AUC	Asymptotic 95% CI		Standard error	*P*-Value	Youden index	Sensitivity (%)	Specificit*y* (%)	Optimal cutoff value
		Lower limit	Upper limit						
NLR	0.841	0.678	1.000	0.083	<0.001	0.7692	76.92	100.00	3.96
NT-proBNP	0.705	0.502	0.907	0.103	0.029	0.5260	76.92	75.68	3815.42 (pg/ml)

## Data Availability

The data can be obtained from the author upon reasonable request.
